# The H_2_S Donor NaHS Changes the Expression Pattern of H_2_S-Producing Enzymes after Myocardial Infarction

**DOI:** 10.1155/2016/6492469

**Published:** 2016-01-05

**Authors:** Na Li, Ming-Jie Wang, Sheng Jin, Ya-Dan Bai, Cui-Lan Hou, Fen-Fen Ma, Xing-Hui Li, Yi-Chun Zhu

**Affiliations:** ^1^Shanghai Key Laboratory of Bioactive Small Molecules, Research Center on Aging and Medicine, Department of Physiology and Pathophysiology, Shanghai Medical College, Fudan University, Shanghai 200032, China; ^2^Center for Developmental Cardiology, Institute for Translational Medicine, College of Medicine, Qingdao University, Qingdao 266021, China; ^3^Department of Physiology, Hebei Medical University, Hebei 050017, China; ^4^Department of Pharmacology, School of Pharmacy, Fudan University, Shanghai 201203, China

## Abstract

*Aims*. To examine the expression patterns of hydrogen sulphide- (H_2_S-) producing enzymes in ischaemic heart tissue and plasma levels of H_2_S after 2 weeks of NaHS treatment after myocardial infarction (MI) and to clarify the role of endogenous H_2_S in the MI process.* Results*. After MI surgery, 2 weeks of treatment with the H_2_S donor NaHS alleviated ischaemic injury. Meanwhile, in ischemia myocardium, three H_2_S-producing enzymes, cystathionine *γ*-lyase (CSE), cystathionine-*β*-synthase (CBS), and 3-mercaptopyruvate sulfurtransferase (3-MST) significantly increased. Plasma H_2_S levels were also elevated.* In vitro*, NaHS treatment protected cardiomyocytes from hypoxic injury and raised CBS levels in a concentration-dependent manner. Different from* in vivo* results, however, CSE or 3-MST expression did not change. NaHS treatment increased the activity of CSE/CBS but not of 3-MST. When CSE was either knocked down (*in vitro*) or knocked out (*in vivo*), H_2_S levels significantly decreased, which subsequently exacerbated the ischaemic injury. Meanwhile, the expressions of CBS and 3-MST increased due to compensation.* Conclusions*. Exogenous H_2_S treatment changed the expressions of three H_2_S-producing enzymes and H_2_S levels after MI, suggesting a new and indirect regulatory mechanism for H_2_S production and its contribution to cardiac protection. Endogenous H_2_S plays an important role in protecting ischaemic tissue after MI.

## 1. Introduction

Hydrogen sulphide (H_2_S) has been recognized as the third gasotransmitter, following nitric oxide and carbon monoxide. It is synthesized endogenously by the catalysis of two pyridoxal-5-phosphate-dependent enzymes, namely, cystathionine-*β*-synthase (CBS) and cystathionine *γ*-lyase (CSE), both utilizing l-cysteine as substrate [1, 2]. CBS is mainly localized in the nervous system, whereas CSE has a crucial role in maintaining cardiovascular homeostasis [3, 4]. The third H_2_S-producing enzyme, 3-mercaptopyruvate sulfurtransferase (3-MST), has recently been discovered; this enzyme generates H_2_S in both the nervous and cardiovascular systems [5]. Accumulating evidence indicates that H_2_S is vital in regulating cardiovascular functions [6]. H_2_S can relax smooth muscle cells by activating ATP-dependent potassium (K^+^) channels (K_ATP_), leading to a subsequent decrease in blood pressure [7]. It also has a substantial role in regulating cellular metabolism and alleviating heart fibrosis and inflammation [8]. H_2_S can reduce infarct size and preserve left ventricular function after MI or myocardial ischaemia/reperfusion* in vivo* [9–11]. It also regulates the outward K^+^ current (Ito) channels, extends action potential duration in epicardial myocytes, and shows efficacious protection against fatal arrhythmias in a rat model of myocardial infarction (MI) [12].

Qipshidze et al. reported that H_2_S promotes angiogenesis and significantly limits the extent of MI injury. They also observed a decrease in CSE expression after MI. NaHS treatment for 4 weeks upregulates CSE but not CBS expression [13]. Zhu et al. also reported the reduction of CSE mRNA in rats 48 h after MI [9]. However, less is known about the expression patterns of the three H_2_S-producing enzymes between 48 h and 4 weeks after MI, during which the fate of ischaemic cardiomyocytes is determined by many endogenous and exogenous signals. In this study, we tested the expressions of three H_2_S-producing enzymes in ischaemic heart tissues 2 weeks after MI and measured plasma H_2_S levels. We also clarified the role of endogenous H_2_S after MI.

## 2. Materials and Methods

### 2.1. The Mouse MI Model and NaHS Administration* In Vivo*

Adult male C57BL/6 mice (8 weeks) were purchased from the Institute of Laboratory Animal Science of the Chinese Academy of Medical Sciences (Shanghai, China). Experimental protocols were approved by the ethics committee for experimental research, Shanghai Medical College, Fudan University.

Mice were anaesthetized and ventilated with a rodent ventilator (Kent Scientific Corporation, USA). A parasternal incision was made with surgical scissors by cutting the skin and intercostal muscles between the left third and fourth ribs; MI was induced by occluding the left anterior descending coronary artery (LAD) using a 7-0 silk suture beneath the LAD, 1 mm inferior to the left auricle. The sham group experienced the same procedure without coronary artery occlusion.

After MI surgery, different concentrations of NaHS solution (0, 25, 50, and 100 *μ*mol/kg/day) were injected intraperitoneally for 2 weeks (first administration was shortly after MI on day 1). Normal saline was used as control. The sham group received same NaHS or normal saline treatment as MI groups. On the 15th day (no NaHS treatment on that day), mice were sent to get echocardiographic assessment. After that mice were anesthetized and killed for plasma to measure H_2_S levels and for protein from ischemic area used for western blot to test the changes of three enzymes.

For acute infarct size determination, NaHS solution (0, 25, 50, and 100 *μ*mol/kg) was administered 15 min before MI surgery. The infarct size is determined on day 2.

### 2.2. Echocardiographic Assessment

Echocardiography was performed as previously described [14]. Briefly, the mice were mildly anaesthetized with isoflurane (1%), and two-dimensional guided M-mode tracings were recorded using a Vevo 770 high-resolution system (Visualsonics, Toronto, Canada). Left ventricular internal dimension systole (LVIDs), left ventricular internal dimension diastole (LVIDd), left ventricular ejection fraction (LVEF), and left ventricular fractional shortening (LVFS) were measured to evaluate left ventricular function. All parameters were the average values from three cardiac cycles.

### 2.3. Determination of Infarct Size

Evans' Blue-2,3,5-triphenyltetrazolium chloride (TTC) double staining was introduced to measure the infarct size and the areas at risk as previously described [10]. Mice were injected with NaHS solution (0, 25, 50, and 100 *μ*mol/kg) for 15 min before MI surgery. Twenty-four hours later, these mice were anaesthetized and their chests were opened again to expose the hearts. Evans' Blue (1.0%, Sigma-Aldrich, St. Louis, MO) solution was injected intravenously into the femoral vein to distinguish ischaemic from nonischaemic areas. The hearts were immediately excised and sliced into 1-2 mm thick slices parallel to the atrioventricular groove and immersed in 1% TTC (Sigma-Aldrich, St. Louis, MO) at 37°C for 15 min. The size of the area at risk (AAR) and the infarct area (INF) were quantified using ImageJ software by an observer blinded to the study.

### 2.4. Western Blot

Proteins were extracted from mouse left ventricles 2 weeks after MI or from cardiomyocytes pretreated with NaHS or vehicle 30 min before the 6 h exposure to hypoxic or normoxic conditions. Protein concentrations were determined by the BCA method (Shen Neng Bo Cai Corporation, Shanghai, China). Protein samples (50 *μ*g) were subjected to 10% SDS-PAGE, transferred to polyvinylidene fluoride membranes (Millipore-Upstate, Billerica, MA, USA), and blocked with 5% nonfat milk. The membranes were then probed with primary antibodies against CSE, CBS (Abcam, Cambridge, UK), or 3-MST (Santa Cruz Biotechnology, CA). GAPDH was used as the internal control (Cell Signaling Technology). These experiments were performed at 4°C overnight. After washing with TBST 3X, the membranes were incubated with horseradish peroxidase-conjugated secondary antibodies at room temperature for 2 h. SuperSignal West Pico Chemiluminescent Substrate (Thermo Scientific-Pierce, Waltham, MA, USA) was then added and detected on radiographic films. Gray values of bands were quantified with the SmartViewer software.

### 2.5. Measurement of H_2_S Levels and the Activity of H_2_S-Producing Enzymes

Whole blood sample was collected, anticoagulated, and centrifuged at 3000 rpm for 15 min to obtain the plasma. The medium from cardiomyocyte cultures was collected. H_2_S levels in plasma or culture medium were measured as previously described [15]. H_2_S levels were calculated using a standard curve generated from a sodium sulphide solution (0–100 *μ*M). The activities of CSE/CBS and 3-MST were measured according to the methods described by Tao et al. [16]. Briefly, cardiomyocytes were incubated with the substrate, l-cysteine, in the presence of pyridoxal-5′-phosphate for CSE/CBS or *α*-ketoglutarate for 3-MST. H_2_S levels were measured, and the amount of H_2_S produced by 1 *μ*g protein/min was calculated, representing the activity of H_2_S-producing enzymes. However, because the detection of CSE and CBS activity shared the same reaction system, their activities could not be separated using this method.

### 2.6. Cell Culture and Treatment

Primary cultures of neonatal cardiomyocytes were established according to previously described methods [10]. The experimental protocol was approved by the ethics committee for experimental research, Shanghai Medical College, Fudan University. In brief, the hearts dissected from 1-day-old Sprague-Dawley rats were washed in cold phosphate-buffered saline (PBS) containing 130 mM NaCl, 3 mM KCl, 1 mM NaH_2_PO_4_, 4 mM glucose, and 20 mM HEPES (pH adjusted to 7.4 with NaOH) for three times to remove blood. The hearts were then minced in a drop of 0.125% trypsin (Sigma-Aldrich, St. Louis, MO, USA) to as small a size as possible and then subjected to a series of incubations at 37°C in a normal saline-buffered trypsin solution. After centrifugation, cell pellets were resuspended in Dulbecco's modified Eagle medium/F-12 (Gibco, Grand Island, NY) containing 10% heat-inactivated fatal bovine serum (Gibco, Grand Island, NY), 100 U/mL penicillin, and 100 *μ*g/mL streptomycin. To increase the purity of cardiomyocytes, dissociated cells were plated in 100 mm culture dishes and kept in a 5% CO_2_ incubator at 37°C for 1 h. Nonmyocytes readily attached to the bottom of the dish, whereas most cardiomyocytes remained suspended in the medium. The resulting suspensions of cardiomyocytes were diluted to a density of 1 × 10^6^ cells/mL and plated in 60 mm dishes or 6-well plates for protein extraction or 96-well plates for the Cell Counting Kit 8 (CCK8) and lactic dehydrogenase (LDH) tests and then cultured in a humidified 5% CO_2_ incubator at 37°C. 5-Bromo-2′-deoxyuridine (100 *μ*M) was added during the first 48 h to prevent proliferation of residual nonmyocytes.

To establish the hypoxia model, cardiomyocytes were cultured in DMEM/F-12 without serum and exposed to hypoxic conditions (95% N_2 _+ 5% CO_2_) for 6 h. For the NaHS treatment groups, 25, 50, and 100 *μ*M of NaHS solution were added 30 min before hypoxia.

CSE small interfering RNAs (CSE siRNA) were purchased from Ambion (Austin, TX, USA). Cardiomyocytes were transfected with 25 nM CSE siRNA using Lipofectamine 2000 (Invitrogen) according to the manufacturer's guidelines.

### 2.7. CCK8 and LDH Activity

Cardiomyocytes were seeded on 96-well plate and treated with vehicle or NaHS for 30 min, followed by 6 h exposure to hypoxic or normoxic conditions. Culture medium was collected and LDH activity was tested according to manufacturer's instructions (Nanjing Jiancheng Bioengineering Institute, Nanjing, China). Cardiomyocytes were used for CCK8 activity measurement according to manufacturer's instructions (Dojindo Molecular Technologies, Japan).

### 2.8. CSE Knock-Out Mice Identification

PCR-genotyping of CSE KO mice was identified according to the methods before [17]. Briefly, genomic DNA was extracted from heart tissues and subjected to PCR with paired primers: CSE knock-out mice (CSE KO) forward, 5′-CCTGGATATAAGCGCCAAAG-3′, and reverse, 5′-AGGAACCAGGGCGTATCTCT-3′, wild type (WT) forward, 5′-CCTGGATATAAGCGCCAAAG-3′, and reverse, 5′-CGAGAATTCCATTGCTCAGG. The amplified DNAs were then identified by DNA electrophoresis, from the representative photo of which we could separate CSE KO mice (single band, 309 bp) from WT mice (single band, 167 bp).

### 2.9. Statistical Analysis

Data are expressed as means ± SEM. Statistical analysis was performed using an SPSS software package, version 17.0 (SPSS, Inc., Chicago, IL, USA). The statistical comparisons among groups were performed by one-way ANOVA. Paired data were evaluated by two-tailed Student's *t*-test. *P* < 0.05 was considered statistically significant.

## 3. Results

### 3.1. The H_2_S Donor (NaHS) Protected Ischaemic Myocardium from Myocardial Infarction Injury

We used echocardiography to evaluate systolic and diastolic function. Echocardiography revealed that 2 weeks of NaHS treatment at 50 and 100 *μ*mol/kg/day significantly increased cardiac function compared with cardiac function after treatment with normal saline. LVEF and LVFS increased, whereas LVIDs and LVIDd decreased (Figures 1(a) and 1(b)). Further, the infarct size was measured by Evans' Blue-TTC staining. NaHS pretreatment at 50 and 100 *μ*mol/kg for 15 min significantly decreased the INF compared with the normal saline group (Figure 1(c)).

The above results showed that NaHS treatment after MI surgery could efficiently protect the ischaemic heart compared with the untreated group.

### 3.2. H_2_S Levels and Expressions of H_2_S-Producing Enzymes Increased with NaHS Treatments

Ischaemic heart tissues from MI mice showed decreased CSE and 3-MST levels after 2 weeks; in contrast, CBS expression significantly increased. Two weeks of NaHS treatments in the range of 25–100 *μ*mol/kg/d significantly increased the protein expression of all three enzymes in ischemia myocardium (Figures 2(a) and 2(c)). In noninfarcted control hearts, NaHS treatment for 2 weeks increased the expression of CSE (50 *μ*mol/kg/day) and 3-MST (25 *μ*mol/kg/day), while NaHS (25–100 *μ*mol/kg/day) did not change expression of CBS (Figure 2(b)). Plasma H_2_S levels decreased after MI surgery, whereas 2 weeks of NaHS treatments alleviated the reduction. NaHS treatment (50 and 100 *μ*mol/kg/day) significantly raised the plasma H_2_S levels after MI (Figure 2(d)).

### 3.3. The H_2_S Donor NaHS Protected Cardiomyocytes from Hypoxia-Induced Injury* In Vitro*

Cardiomyocytes are the major heart cells, and more importantly, they are highly terminated and cannot proliferate after birth. Protecting cardiomyocytes from ischaemic injury is essential. LDH and CCK8 tests are classic methods to detect cell viability and toxicity. Compared with the normoxic group, LDH activity in the culture medium of cardiomyocytes exposed to hypoxic conditions was much higher, whereas NaHS treatment in the range of 25–100 *μ*M significantly decreased LDH activity. NaHS treatment at 50 and 100 *μ*M also increased CCK8 values, indicating improved cardiomyocyte activity (Figure 3(a)). Cells produced less H_2_S under hypoxic conditions, whereas NaHS treatment significantly increased H_2_S production in a concentration-dependent manner (Figure 3(b)). Different from the enzyme expression patterns in ischaemic heart tissues, hypoxia did not change CSE or 3-MST expressions, whereas an increase in CBS expression still occurred* in vitro*. NaHS treatments did not change CSE or 3-MST expressions under hypoxic conditions but caused an increase in CBS levels in a concentration-dependent manner (Figures 3(c) and 3(d)). Hypoxia decreased the activity of CSE/CBS, and 50 *μ*M NaHS treatment significantly diminished this decrease (Figure 3(e)). 3-MST activity was not influenced (Figure 3(f)).

### 3.4. Endogenous H_2_S Protected Ischaemic Myocardium from Myocardial Infarction Injury

CSE is the main H_2_S-producing enzyme in the cardiovascular system, catalyzing the synthesis of endogenous H_2_S from l-cysteine; we used CSE KO mice to study whether endogenous H_2_S plays a role in cardiac protection after MI. CSE KO mice were characterized by analysing genomic DNA, CSE mRNA, and protein levels, which were compared with WT mice (Figure 4(a)). Plasma H_2_S levels in four groups were then tested: (1) CSE KO without MI, (2) CSE KO with MI, (3) WT without MI, and (4) WT with MI. As expected, plasma H_2_S levels were significantly lower in mice from the CSE KO without MI group than from the WT without MI group. Plasma H_2_S levels decreased significantly after MI both in WT and in CSE KO groups (Figure 4(b)). Furthermore, as shown in Figure 4(c), INFs in CSE KO mice were more extensive than those in WT mice. Protein expression of the other two enzymes, CBS and 3-MST, increased in CSE KO mice, most likely due to compensation (Figure 4(d)).

### 3.5. Endogenous H_2_S Protected Cardiomyocytes from Hypoxia-Induced Injury

We used CSE siRNA to knockdown CSE expression and then monitored H_2_S levels in the culture medium. Compared with the hypoxia control, addition of CSE siRNA caused a significant decrease in H_2_S levels in culture medium and CSE expression in cardiomyocytes. The expressions of CBS and 3-MST in cardiomyocytes significantly increased after adding CSE siRNA (Figures 5(a) and 5(b)). The activity of the three H_2_S-producing enzymes did not change after the addition of CSE siRNA (Figure 5(c)). Cardiomyocyte injury was also evaluated after the addition of CSE siRNA. LDH activity was increased and CCK8 values were decreased, suggesting that knockdown of CSE expression exacerbated hypoxic injury (Figure 5(d)).

## 4. Discussion

In this study, we used an* in vivo* MI model and an* in vitro* hypoxic cardiomyocyte model to systemically investigate the regulation of exogenous H_2_S on the expression of the three H_2_S-producing enzymes. CSE KO mice were also used to study the effect of endogenous H_2_S on the ischaemic hearts. Cardiac expressions of the three enzymes were quantified 2 weeks after MI surgery. Our experiments indicated four important findings: (1) exogenous H_2_S significantly increased the expression of the three enzymes* in vivo*, (2) 25–100 *μ*M NaHS pretreatment increased CBS levels in a concentration-dependent manner, and 50 *μ*M NaHS treatment increased CSE/CBS activity* in vitro*, (3) endogenous H_2_S played an important role in protecting the ischaemic heart after MI, and (4) when CSE was either knocked down (*in vitro*) or knocked out (*in vivo*), the expressions of CBS and 3-MST increased due to compensation.

Accumulating evidence has confirmed that H_2_S is vital in regulating cardiovascular functions. H_2_S can relax smooth muscle cells by activating ATP-dependent K^+^ channels (K_ATP_), leading to a subsequent decrease in blood pressure [7]. H_2_S reduces infarct size and preserves left ventricular function after MI or myocardial ischemia/reperfusion [9–11]. In this study, we used echocardiography and Evans' Blue-TTC double staining to detect the protective role of 2-week H_2_S treatment to mice suffering from MI injury. NaHS treatment at 50 and 100 *μ*mol/kg after MI surgery effectively protected the heart from ischaemic damage. This protection was accompanied by greater CSE and 3-MST expression. From our results in Figure 3(c) those NaHS treatments did not change CSE or 3-MST expression under hypoxic condition* in vitro*; the elevated CSE and 3-MST expression after myocardial infarction by NaHS treatment* in vivo* is likely resulting from the improvement of cardiac function (e.g., less overload of noninfarcted area in NaHS-treated animals), but not from direct effect of H_2_S on these enzymes.

The mechanisms in which exogenous H_2_S participates in cardiac protection have been studied for years but still are not completely clear. H_2_S promotes the secretion of proangiogenic factors, such as VEGF, which appears to enhance angiogenesis in the ischaemic heart and improve blood supply [13, 18]. Inhibition of cardiomyocyte apoptosis also appears to play an important role in H_2_S-mediated cardiac protection [10, 11]. Recently, King reported eNOS-dependent cytoprotection by H_2_S in the setting of I/R injury [19]. The manner in which exogenous H_2_S affects another gaseous signalling molecule suggests that we should examine whether exogenous H_2_S influences endogenous H_2_S production to protect the ischaemic heart. In this study, we detected H_2_S levels in plasma and H_2_S-producing enzyme expression in the hearts.

After 2 weeks of intraperitoneal injection of NaHS (25–100 *μ*mol/kg/day), the expressions of the three enzymes in ischemia myocardium increased but to different levels. In noninfarcted myocardium, NaHS treatment for 2 weeks increased the expression of CSE (50 *μ*mol/kg/day) and 3-MST (25 *μ*mol/kg/day), while NaHS (25–100 *μ*mol/kg/day) did not change expression of CBS. Our results suggested that both myocardial infarction surgery (Figure 2(a)) and exogenous NaHS administration (Figures 2(b) and 2(c)) influenced the expression of H_2_S-synthesizing enzymes in infarcted hearts. ① Myocardial infarction decreased the CSE expression, while exogenous NaHS administration increased its expression. The overall effect of exogenous NaHS administration on CSE in infarcted heart was elevation. ② Myocardial infarction increased the CBS expression, while exogenous NaHS administration did not change its expression. The overall effect of exogenous NaHS administration on CBS in infarcted heart was elevation. ③ Myocardial infarction decreased the 3-MST expression, while exogenous NaHS administration increased its expression. The overall effect of exogenous NaHS administration on 3-MST in infarcted heart was elevation. The complicated* in vivo* situations that caused the effect of NaHS on CBS and CSE was not ideally dose-dependent and effect on 3-MST was maximal at 50 *μ*mol/kg. NaHS treatment at 50 and 100 *μ*mol/kg/day significantly increased plasma H_2_S levels. Qipshidze et al. previously reported that the expression of CSE increased and CBS decreased after drinking an H_2_S-releasing aqueous solution for 4 weeks [13]. The possible explanation for the different results between Qipshidze et al.'s study and ours could be the different duration of NaHS treatment; 2 weeks was used in the present study, whereas Qipshidze et al.'s research extended to 4 weeks. Changes in plasma H_2_S levels might also affect the expressions of the three enzymes.

Cardiomyocytes are the major cell type in the heart. We next investigated whether H_2_S could protect cardiomyocytes from hypoxia-induced injury* in vitro*. Similar to the* in vivo* results, H_2_S protected cardiomyocytes from hypoxic injury, as was evidenced by lower LDH activity in the culture medium and higher cellular CCK8 values. Simultaneously, H_2_S levels in NaHS-treated groups significantly increased. Because the expression and activity of both enzymes contribute to H_2_S production, we next tested the expression as well as the activity of the three enzymes. While the expressions of CSE or 3-MST did not change, CBS expression increased in a concentration-dependent manner. Hypoxia decreased the activity of CSE/CBS without affecting 3-MST, which may have contributed to the decrease in H_2_S levels under hypoxic conditions. Similarly, NaHS treatment may increase the activity of CSE/CBS to produce more H_2_S.

The difference between* in vivo* (H_2_S enhanced the expression of all three enzymes) and* in vitro* (H_2_S only enhanced the expression of CBS) studies may be due to the fact that the heart contains several kinds of cells and that H_2_S can be synthesized in cells other than cardiomyocytes. CSE, the major H_2_S-producing enzyme in cardiovascular systems, is also expressed in smooth muscle cells [7, 19], and 3-MST also exists in endothelial cells [5]. Cells surrounding cardiomyocytes can release H_2_S to maintain local H_2_S concentrations. Exogenous H_2_S can change the expressions of H_2_S-producing enzymes in other cell types. For example, Na_2_S (another H_2_S donor) also enhances CSE expression in ischemia/reperfusion-stimulated brain endothelial cells [20]. Results from tissue samples revealed overall H_2_S production, not just that from cardiomyocytes.

The mechanisms of upregulation of CBS by exogenous H_2_S need to be studied in the future. Exogenous H_2_S could specifically increase CBS expression with no effect on CSE or 3-MST, which might elevate local H_2_S concentrations and thus result in cardiac protection for different reasons. Wang et al. reported that exogenous H_2_S (10–80 *μ*M) downregulates CSE expression, whereas hypoxia upregulates CSE expression in mammalian cell lines [21, 22]; these results differed from those obtained in the study. The probable explanation is that they used cell lines and NaHS treatment or hypoxia was administered separately. In our experimental conditions, we used primary cardiomyocytes and studied H_2_S effects under hypoxic conditions (a combination of hypoxia and NaHS treatment), which better mimicked post-MI conditions; this may reveal the mechanism of cardiac protection of H_2_S.

Finally, we used CSE KO mice or CSE siRNA to study the protective role of endogenous H_2_S. When CSE was either knocked out* in vivo* or knocked down* in vitro*, the ischaemic heart or cardiomyocytes displayed more damage; at the same time, although CBS and 3-MST expression increased due to compensation, H_2_S concentration still significantly decreased, confirming that CSE is the main H_2_S-producing enzyme in the heart. In cardiomyocytes, CSE siRNA significantly decreased CSE protein levels, but the activity of the three enzymes did not change. Low H_2_S levels in the medium may be the result of decreased CSE protein expression. In another study, King et al. also showed that CSE KO mice had large INFs, and the infarct size became less extensive when exogenous H_2_S was added [19]. King's experiments also confirmed that sufficient local H_2_S production around ischaemic tissues appears to be important for cardioprotection. When the major H_2_S-producing enzyme did not function adequately, H_2_S levels dropped and the protective effects of H_2_S were impaired.

## 5. Conclusion

In summary, we demonstrated for the first time that 2 weeks of exogenous H_2_S treatment can increase the expression of the three H_2_S-producing enzymes in ischaemic heart tissue and alleviate ischaemic damage. Endogenous H_2_S also appears to have a major role in protecting the ischaemic heart. This study suggested a new and indirect regulatory pathway for cardiac protection; however, the underlying mechanism needs further investigation.

## Figures and Tables

**Figure 1:** The H_2_S donor NaHS protects ischaemic myocardium from myocardial infarction injury. (a) Representative echocardiogram from the sham, MI surgery control, and NaHS 50 *μ*mol/kg/day treatment groups; (b) Echocardiographic parameter analysis. LVEF, left ventricular ejection fraction; LVFS, left ventricular fractional shortening; LVIDs, left ventricular internal dimension systole; LVIDd, left ventricular internal dimension diastole. (c) Statistics of Evans' Blue-TTC staining to show the percentage of area at risk or infarct area. LV, left ventricle; AAR, area at risk; and INF, infarct area. Numbers inside bars denote the number of animals per group. Values are mean ± SE. ^*∗*^ *P* < 0.05 and ^*∗∗*^ *P* < 0.01.

**Figure 2:** Exogenous H_2_S increased plasma H_2_S levels and the three H_2_S-producing enzymes expression in ischaemic myocardium. (a) The expressions of CSE and 3-MST significantly decreased, whereas CBS expression increased 2 weeks after MI surgery. (b) In noninfarcted myocardium, NaHS treatment for 2 weeks increased the expression of CSE (50 *μ*mol/kg/day) and 3-MST (25 *μ*mol/kg/day), while NaHS (25–100 *μ*mol/kg/day) did not change expression of CBS; (c) H_2_S donor NaHS (25–100 *μ*mol/kg/day) increased the expression of the three enzymes in ischaemic myocardium 2 weeks after MI. (d) Changes in plasma H_2_S levels in sham, MI surgery control, and NaHS treatment groups. Plasma H_2_S levels decreased 2 weeks after MI, whereas 50 and 100 *μ*mol/kg/day NaHS treatment ameliorated this trend. Numbers inside bars denote the number of animals per group. Values are mean ± SE. ^*∗*^ *P* < 0.05.

**Figure 3:** H_2_S donor NaHS protects cardiomyocytes from hypoxia-induced injury. (a) Cell viability was detected with LDH and CCK8 kits. Hypoxia exposure decreased cell viability, as evidenced by high LDH activity and low CCK8 values; 30 min of NaHS pretreatment alleviated the above injury, as demonstrated by the significant drop in LDH activity and increase in CCK8 values; (b) H_2_S level in the culture medium decreased after exposure to hypoxia, and 25–100 *μ*M NaHS pretreatment in a concentration-dependent manner caused elevation of H_2_S levels; (c) 6 h hypoxia exposure did not change CSE or 3-MST expressions but significantly increased CBS expression; (d) NaHS pretreatment did not change the expression of either CSE or 3-MST but increased CBS expression at 100 *μ*M. (e) The activity of CSE/CBS declined after exposure to hypoxia, whereas 50 *μ*M NaHS treatment caused a significant increase in their activity; (f) Hypoxia with or without NaHS treatment did not change the activity of 3-MST. Numbers inside bars denote the number of animals per group. Values are mean ± SE. ^*∗*^ *P* < 0.05 and ^*∗∗*^ *P* < 0.01.

**Figure 4:** Endogenous H_2_S protected ischaemic myocardium from myocardial infarction injury. (a) Characterization of CSE knock-out mice (CSE KO). Left panel: PCR analysis of genomic DNA from CSE KO mice and wide type mice (WT). Middle panel: real-time PCR analysis of CSE mRNA expression in the hearts from WT and CSE KO mice; right panel: representative western blot of CSE protein expression. (b) Plasma H_2_S levels in WT and CSE KO mice with (MI) or without (sham) surgery. Plasma H_2_S levels from the highest to lowest were as follows: WT without surgery, CSE KO without surgery, WT with MI surgery, and CSE KO with MI surgery; (c) infarct area in CSE KO group was larger than that in WT group detected with Evans' Blue-TTC staining; (d) expression of CBS and 3-MST increased in CSE KO mice. Numbers inside bars denote the number of animals per group. Values are mean ± SE. ^*∗*^ *P* < 0.05 and ^*∗∗*^ *P* < 0.01.

**Figure 5:** Endogenous H_2_S protected cardiomyocytes from hypoxia-induced injury. (a and b) Compared with the hypoxia control, CSE siRNA significantly decreased CSE expression and H_2_S levels in the culture medium, whereas CBS and 3-MST expressions increased; (c) the activity of the three H_2_S-producing enzymes did not change after CSE siRNA treatment. (d) CSE siRNA exacerbated hypoxia injury, demonstrated by an increase in LDH activity and a decrease in CCK8 values. Numbers inside bars denote the number of animals per group. Values are mean ± SE. ^*∗*^ *P* < 0.05 and ^*∗∗*^ *P* < 0.01.
